# Neuroimaging Correlates of Resilience to Traumatic Events—A Comprehensive Review

**DOI:** 10.3389/fpsyt.2018.00693

**Published:** 2018-12-12

**Authors:** Julia Bolsinger, Erich Seifritz, Birgit Kleim, Andrei Manoliu

**Affiliations:** ^1^Department of Psychiatry, Psychotherapy and Psychosomatics, Psychiatric University Hospital, University of Zurich, Zurich, Switzerland; ^2^Department of Psychology, University of Zurich, Zurich, Switzerland

**Keywords:** resilience, trauma, PTSD, magnetic resonance imaging, neuroimaging

## Abstract

Improved understanding of the neurobiological correlates of resilience would be an important step toward recognizing individuals at risk of developing post-traumatic stress disorder (PTSD) or other trauma-related diseases, enabling both preventative measures and individually tailored therapeutic approaches. Studies on vulnerability factors allow drawing conclusions on resilience. Structural changes of cortical and subcortical structures, as well as alterations in functional connectivity and functional activity, have been demonstrated to occur in individuals with PTSD symptoms. Relevant areas of interest are hippocampus, amygdala, insula, anterior cingulate cortex, and prefrontal cortex, as well as related brain networks, such as the default-mode, salience, and central executive network. This review summarizes the existing literature and integrates findings from cross-sectional study designs with two-group designs (trauma exposed individuals with and without PTSD), three-group designs (with an additional group of unexposed, healthy controls), twin-studies and longitudinal studies. In terms of structural findings, decreased hippocampal volume in PTSD individuals might be either a vulnerability factor or a result of trauma exposure, or both. Reduced anterior cingulate cortex and prefrontal cortex volumes seem to be predisposing factors for increased vulnerability. Regarding functional connectivity, increased amygdala connectivity has been demonstrated selectively in PTSD individuals, as well as increased default-mode-network and salience network connectivity. In terms of functional activity, increased amygdala and anterior cingulate cortex activities, and decreased prefrontal cortex activity as a response to external stimuli have been associated with higher vulnerability. Increased prefrontal cortex activity seemed to be a protective factor. Selecting adequate study designs, optimizing the diagnostic criteria, as well as differentiating between types of trauma and accounting for other factors, such as gender-specific differences, would be well-served in future research. Conclusions on potential preventative measures, as well as clinical applications, can be drawn from the present literature, but more studies are needed.

## Introduction

Over the past decade, psychiatric, psychological and neurobiological research has increasingly focused on the phenomenon of resilience, which is conceptualized as the ability to maintain a normal, i.e., pre-trauma level of functioning and avoid deteriorating mental disorders, even after experiencing extreme stress or trauma (1). The term resilience does not describe a static component, but rather a dynamic adaptive process that involves cognition and/or emotion regulation, ultimately resulting in functional coping mechanisms (2). Consequently, a better understanding of the neurobiological underpinnings of involved dynamic neurocognitive processes might contribute to a better operationalization and understanding of the concept of resilience (3).

Traditionally, research on resilience focused on the identification of empirical behavioral parameters predictive of the outcome of coping strategies (4). To date, research has mainly focused on identification of neuronal mechanisms associated with greater vulnerability for the development of stress-associated psychiatric diseases, such as post-traumatic stress disorder (PTSD). Identification of such mechanisms are not just the flipside of resilience, but they may lead to a better understanding of the neurobiological correlates of resilience.

In general, specific cerebral structures have been demonstrated to play a crucial role in processing stimuli, as well as in generating reactions to stressors, both in healthy individuals and in patients with psychiatric disease following exposure to trauma. Structural changes of both cortical and subcortical areas have been described, with a particular relevance of hippocampus, amygdala, insular cortex, anterior cingulate cortex (ACC), and medial prefrontal cortex (PFC, see also Figure 1 for a corresponding graphical presentation of relevant neuroanatomical structures) (5). Volume reduction of the hippocampus, a structure of core importance for declarative memory and for regulative processes via the hypothalamic-pituitary-adrenal axis (6), has been shown to be associated with increased emotional and hormonal reactions to stressors (7), as well as changes in conditioned fear reactions (8). Lesions of the amygdala, a structure capable of releasing stress-associated hormones via activation of the hypothalamic-pituitary-adrenal axis (8), have been shown to significantly affect reactions to negative stimuli (9). The insula plays an important role in the regulation of cognitive control and attention (10), as well as—along with the hippocampus—in processing potential threats (11). Changes in ACC activity have been shown to be associated with altered emotion regulation in affective and anxiety disorders (12). The conventional differentiation between ventral-rostral ACC as a modulator of emotional stimuli and dorsal-caudal ACC as a region associated with non-emotional cognitive processes seems to be mollified in more recent studies (12). The PFC plays a role in mediating higher cognitive functions and in regulating limbic structures, especially the amygdala (13, 14), which has been shown by numerous studies to actively be inhibited by the PFC (15).

**Figure 1:** Discussed neuroanatomical structures. This figure presents neuroanatomical target regions frequently investigated via structural or functional MRI in studies assessing potential neurobiological correlates of vulnerability to stress and/or resilience.

Regarding the fact that resilience is regarded as a dynamic adaptation process, examining its functional neurobiological correlates besides analyzing structural findings is of core relevance. Functional magnetic resonance imaging (fMRI) is gold standard for such studies, allowing not only an analysis of neuronal activity patterns but also of network architecture in terms of interactions between spatially separate brain areas (16). The description of intrinsic brain networks and their reactions to intrinsic and extrinsic stimuli has contributed significantly to an improved understanding of the functional architecture of emotional and cognitive processes (17). Three main networks play a role in these processes: the default-mode-network (DMN), including hippocampus, PFC, precuneus and temporoparietal regions, mediates internally directed processes, such as self-referential cognitive tasks (18). The central executive network (CEN) includes lateralized fronto-parietal regions and mediates externally directed processes, such as the modulation of spatial attention (19). The salience network (SN) includes ACC, insula, and amygdala and mediates interaction between DMN and CEN regarding dynamic prioritizing of internal and external stimuli (20). Intrinsic functional connectivity, or the synchronous resting state activity fluctuation, is a surrogate of connectivity within the respective network and according to present knowledge has a high predictive value regarding emotional and cognitive processes in both healthy and mentally ill individuals. Its examination can thus provide a suitable approach to better describe functional correlates of resilience.

Studies involving specific tasks aimed at activating cognitive and/or emotional processes allow to determine the extent of activation for individual brain areas that are recruited during the respective tasks. Comparisons can thus be made between group-specific activity patterns as reactions to external stimuli (21).

The present state of trauma and vulnerability literature is critically reflected with regards to the above aspects, taking into consideration findings on structural changes, functional connectivity and functional activity. Traumatic events include war, natural catastrophes, physical/sexual abuse, or severe accidents. While a direct inverse relationship between resilience and vulnerability does not exist, drawing conclusions from vulnerability studies seems to present the best available approximation to the concept of resilience from a modern imaging point of view at present.

## Review of the Current Literature

Which types of fMRI studies are needed in order to draw meaningful conclusions about resilience in the context of trauma? Selecting a suitable study design is a great challenge of conducting scientific research into the concept of resilience. In order to determine structural and/or functional parameters predicting the development of PTSD following a traumatic event, recruiting study participants *before* their experiencing a trauma would be the desired approach. Comparing subjects developing clinically relevant PTSD symptoms to those proving resilient later, as well as taking into account the dynamic adaptation process inherent in the concept of resilience, would then enable the retrospective identification of such parameters (22). Since such a design is difficult to embrace for logistical reasons, present approaches include cross-sectional study designs with two-group designs (trauma exposed individuals with and without PTSD), three-group designs (with an additional group of unexposed, healthy controls), twin-studies and longitudinal studies.

Since the aim of the current review is to discuss potential structural or functional correlates of vulnerability/resilience to stress, literature research was conducted according to van der Werff and colleagues (22). Studies available by December 2017 were searched in the databases of PubMed at the National Library of Medicine, using the search terms proposed by van der Werff and colleagues, resulting in 45 studies explicitly investigating potential correlates of resilience as assessed via neuroimaging. In the following section, the identified studies are discussed with regards to structural changes, functional connectivity, and functional activity of relevant brain regions that distinguish resilient individuals from those who succumb to trauma and develop PTSD or other trauma-related disorders (see also Tables 1–**3** for detailed presentation of discussed studies).

**Table 1:** Summary of structural findings.

**Authors**	**Study design**	**PTSD**			**TENP**			**HC**			**Results**
		***N***	**M/F**	**Age**	***N***	**M/F**	**Age**	**N**	**M/F**	**Age**	
**HIPPOCAMPUS**											
Lindauer et al. (24)	2 groups	14	8/6	35.4 ± 11.2	14	8/6	36.9 ± 10.1	None			Decreased in PTSD
Lindauer et al. (25)	2 groups	18	8/10	39.6 ± 9.0	14	8/6	36.9 ± 10.1	None			No effect of psychotherapy
Chen et al. (26)	2 groups	12	8/4	34.56 ± 4.91	12	8/4	33.25 ± 5.27	None			Decreased in PTSD
Woodward et al. (32)	2 groups	51	38M	53.5 ± 2.6	48	25M	56.0 ± 3.5	None			Decreased in PTSD, but possibly associated with comorbid alcohol use disorder
Yehuda et al. (31)	2 groups	17	17M	60.6 ± 7.0	16	16M	65.1 ± 9.9	None			No effect, but selectively decreased in individuals with immediate onset PTSD
Felmingham et al. (29)	2 groups	21	NR	NR	17	NR	NR	None			Associated with duration of symptoms
Rogers et al. (30)	2 groups	9	5/4	44.56 ± 15.96	16	10/6	44.44 ± 1 3.60	None			No effect
Wang et al. (33)	2 groups	17	17M	41.0 ± 12.0	19	19M	38.0 ± 15.0	None			Only specific subregions decreased in PTSD
Zhang et al. (28)	2 groups	10	10	40.80 ± 6.83	10	10M	34.30 ± 5.37	None			Decreased in PTSD
Morey et al. (27)	2 groups	99	79/20	38.4 ± 9.9	102	86/16	37.5 ± 10.6	None			Decreased in PTSD
Gurvits et al. (46)	3 groups	7	7M	44.4 ± 1.7	7	7M	47.6 ± 2.9	8	8M	38.1 ± 10.0	Selectively decreased in PTSD, correlated with duration of trauma-exposure
Fennema-Notestine et al. (50)	3 groups	11	11F	33.5 ± 10.3	11	11F	35.4 ± 9.6	17	17F	35.3 ± 12.5	No effect
Bremner et al. (47)	3 groups	10	10F	35.0 ± 6.0	12	12F	32.0 ± 8.0	11	11F	38.0 ± 7.0	Strong decrease in PTSD, moderate decrease in TENP
Pederson et al. (51)	3 groups	17	17F	24.8 ± 5.2	17	17F	26.8 ± 6.6	17	17F	23.8 ± 5.6	No effect
Winter and Irle (49)	3 groups	15	15M	42.0 ± 10.0	15	15M	41.0 ± 11.0	15	15M	41.0 ± 17.0	Correlated with severity of trauma
Golier et al. (53)	3 groups	14	5/9	70.5 ± 5.6	13	6/7	68.5 ± 7.3	20	13/7	71.4 ± 6.4	No effect
Vythilingam et al. (54)	3 groups	14	8/6	35.0 ± 9.0	23	15/8	35.0 ± 7.0	23	9/20	34.0 ± 10.0	Decreased for distinct subregions in PTSD and TENP
Freeman et al. (52)	3 groups	10	10M	79.6 ± 3.2	10	10M	79.8 ± 2.8	6	6M	80.8 ± 3.5	No effect
Apfel et al. (48)	3 groups	41	32/9	42.1 ± 9.6	64	58/6	44.4 ± 9.6	95	81/14	46.4 ± 9.6	Correlated with current symptoms
Morey et al. (55)	3 groups	31	15/16	9.9 ± 2.5	32	15/17	10.0 ± 2.7	57	25/32	10.82 ± 2.5	Increased in TENP
Gilbertson et al. (11)	Twin study	12 (twin pairs)	12M	53.1 ± 3.3	23 (twin pairs)	23M	51.8 ± 2.3	None			Decreased in PTSD paires compared to TENP paires
Pitman et al. (64)	Twin study	25 (twin pairs)	25M	NR	24 (twin pairs)	24M	NR	None			Decreased in PTSD paires compared to TENP paires
Bonne et al. (67)	Longitudinal	10	3/7	33.7 ± 8.9	27	5/12	29.8 ± 10.1	None			No predictor for therapy outcome
Rubin et al. (68)	Longitudinal	Treatment responders/ nonresponders: *n* = 23/17	Responders: 5/18, non-responders: 7/10	Responders: 34.4 ± 8.5/ Non-responders: 37.5 ± 10.7	36	11/25	34.4 ± 10.8	None			Predictor for therapy outcome
**AMYGDALA**											
Lindauer et al. (24)	2 groups	14	8/6	35.4 ± 11.2	14	8/6	36.9 ± 10.1	None			No effect
Lindauer et al. (25)	2 groups	18	8/10	39.6 ± 9.0	14	8/6	36.9 ± 10.1	None			No effect
Rogers et al. (30)	2 groups	9	5/4	44.56 ± 15.96	16	10/6	44.44 ± 13.60	None			No correlation with symptom severity
Kuo et al. (35)	2 groups	42	42M	49.5 ± 8.6	45	45M	44.5 ± 7.3	None			Increased for TENP
Morey et al. (27)	2 groups	99	79/20	38.4 ± 9.9	102	86/16	37.5 ± 10.6	None			Decreased for PTSD
Gurvits et al. (46)	3 groups	7	7M	44.4 ± 1.7	7	7M	47.6 ± 2.9	8	8M	38.1 ± 10.0	No effect
Fennema-Notestine et al. (50)	3 groups	11	11F	33.5 ± 10.3	11	11F	35.4 ± 9.6	17	17F	35.3 ± 12.5	No effect
Morey et al. (55)	3 groups	31	15/16	9.9 ± 2.5	32	15/17	10.0 ± 2.7	57	25/32	10.82 ± 2.5	Selectively increased for TENP
Gilbertson et al. (11)	Twin study	12	12M	53.1 ± 3.3	23	23M	51.8 ± 2.3	None			No effect
Bonne et al. (67)	Longitudinal	10	3/7	33.7 ± 8.9	27	5/12	29.8 ± 10.1	None			No effect
**INSULA**											
Chen et al. (26)	2 groups	12	8/4	34.56 ± 4.91	12	8/4	33.25 ± 5.27	None			Decreased in PTSD
Kasai et al. (65)	Twin study	18 twin pairs	18M	52.8 ± 3.4	23 twin pairs	23M	51.8 ± 2.3	None			Decreased in combat-exposed individuals with PTSD
**ACC**											
Rauch et al. (37)	2 groups	9	9F	51.7 ± 1.9	9	9F	52.0 ± 1.9	None			Decreased (pgACC only) in PTSD
Woodward et al. (32)	2 groups	51	38M	53.5 ± 2.6	48	25M	56.0 ± 3.5	None			Decreased in PTSD
Chen et al. (26)	2 groups	12	8/4	34.56 ± 4.91	12	8/4	33.25 ± 5.27	None			Decreased in PTSD
Felmingham et al. (29)	2 groups	21	NR	NR	17	NR	NR	None			Decreased in PTSD
Rocha-Rego et al. (38)	2 groups	16	7/9	43.3 ± 5.78	16	7/9	44.9 ± 6.60	None			Decreased (pgACC only) in PTSD
Eckart et al. (56)	3 groups	20	20M	36.2 ± 7.7	19	19M	34.1 ± 9.9	13	13M	29.0 ± 7.2	Strong decrease in PTSD, moderate decrease in TENP
Kasai et al. (65)	Twin study	Kasai et al. (65)	18M	52.8 ± 3.4	23 twin pairs	23M	51.8 ± 2.3	None			PTSD diagnosis × combat exposure interaction in pgACC (in which combat-exposed PTSD twins had lower gray matter density than their own combat-unexposed cotwins and TENP-twins)
**PFC**											
Felmingham et al. (29)	2 groups	21	NR	NR	17	NR	NR	None			Decreased in PTSD and TENP
Fennema-Notestine et al. (50)	3 groups	11	11F	33.5 ± 10.3	11	11F	35.4 ± 9.6	17	17F	35.3 ± 12.5	Decreased in PTSD and TENP
Eckart et al. (56)	3 groups	20	20M	36.2 ± 7.7	19	19M	34.1 ± 9.9	13	13M	29.0 ± 7.2	Selectively decreased in PTSD
Morey et al. (55)	3 groups	31	15/16	9.9 ± 2.5	32	15/17	10.0 ± 2.7	57	25/32	10.82 ± 2.5	Selectively decreased in PTSD

*Study design and study sample characteristics are presented for all discussed studies investigating potential correlates of vulnerability/resilience to stress as assessed via structural MRI. PTSD, post-traumatic stress disorder; TENP, trauma-exposed non-PTSD; HC, healthy controls; NR, not reported*.

### Two-Group-Studies

The majority of studies compare in a cross-sectional design individuals who have developed PTSD symptoms after trauma exposure (“PTSD”) to individuals who have not developed such symptoms post-trauma (trauma-exposed-non-PTSD, “TENP”). One major disadvantage of this design is the lack of a non-exposed control group. It can thus not be clearly identified whether findings are due to trauma exposure and the resulting stress, *per se*, or a result of other factors.

#### Structure

In one of the first studies to investigate a potential association between morphological properties of the hippocampus and clinical outcome of trauma, Bremner et al. found that hippocampal volume in veterans with PTSD was reduced compared to healthy, non-exposed controls (23). Lindauer et al. examined the hippocampal volume of 28 policemen following trauma exposure, of which 14 developed PTSD symptoms while 14 remained symptom-free. Bilaterally reduced hippocampal volume was shown in the PTSD group, and a correlation was shown between volume reduction and PTSD severity, especially flashbacks (24). A follow-up study of the same group demonstrated that successful psychotherapy did not influence hippocampal volume (25). Reduced hippocampal volume of PTSD groups compared to healthy controls were also shown in a cohort of 24 burn victims (26), a cohort of 200 war veterans (27), and a cohort of 20 victims in a coal mine flood (28). In addition, the latter study demonstrated a statistical correlation between hippocampal volume reduction and clinical symptom severity. Another study not only confirmed hippocampal volume reduction in PTSD individuals, but also demonstrated a correlation with PTSD symptom duration (29). Contrarily, a study on 25 victims of the Sarin terrorist attack in Tokyo failed to replicate these findings (30). Yehuda et al. found no differences in hippocampal volume between war veterans with or without PTSD symptoms, yet demonstrated a selective reduction of hippocampal volume in individuals developing PTSD symptoms immediately following trauma exposure (31). They also observed a correlation in the PTSD group of hippocampal volume and reduced memory capacity, as well as decreased urine cortisol, which might indicate permanently increased stress levels in affected individuals. Another study including 99 war veterans with or without PTSD symptoms also failed to demonstrate hippocampal volume differences initially, yet selectively observed such a reduction in PTSD patients also diagnosed with an alcohol dependence syndrome (32). Findings of a study in 36 war veterans implicate that volume reduction might be present only in certain hippocampal regions (cornu ammonis 3/dentate gyrus) (33), regions closely associated with neuroneogenesis (34). Regarding the amygdala, 2-group-studies on structural changes present heterogeneous findings. A study on policemen found no differences in amygdala volume between PTSD and TENP groups (24), and these findings were replicated by the same group later (25). A more recent study demonstrated reduced amygdala volume in PTSD individuals, yet did not find a correlation between volume reduction and symptom severity (27). A study on 25 terrorist victims observed both reduced amygdala volume and a correlation between reduction and symptom severity in PTSD individuals (30). Contrarily, yet another study found an increase in amygdala volume in PTSD individuals compared to TENP (35). With respect to the insular cortex, Chen et al. described bilaterally reduced insular volume in burn victims with PTSD compared to TENP (26). Across current literature, the volume of the ACC was consistently reduced in patients with PTSD symptoms compared to TENP individuals. In more detail, Gulf war veterans with PTSD symptoms had significantly reduced ACC volume compared to those without PTSD, even after controlling for other variables, such as alcohol dependence syndrome (36). Studies on 24 burn victims (26) and on 38 traffic accident or mugging victims without further comorbidities (29) confirmed these findings. Studies on Vietnam War nurses (37) and public violence victims (38) found selective volume reductions in pgACC of PTSD individuals compared to TENP, without changes in other ACC areas. Finally, PTSD individuals were found to have significantly reduced superior medial PFC and orbitofrontal gyrus volumes compared to TENP (29, 35).

#### Functional Connectivity

Connectivity between amygdala and insula has been shown to be increased in PTSD individuals (Iraq War veterans) compared to TENP individuals, while there were no between-group differences regarding amygdala-PFC connectivity (39). Increased amygdala-insula connectivity in the PTSD group was also observed in another study on war veterans (40), with the additional finding of decreased amygdala/hippocampus-ACC connectivity. Additionally, a more recent study on war veterans demonstrated increased amygdala-pgACC and amygdala-dorsomedial PFC connectivity in the PTSD group compared to the TENP group (41). Yet another study, using DSM-V diagnostic criteria (unlike the previously quoted studies), found increased connectivity between Amygdala and medial PCF, as well as hippocampus, in the PTSD group (42). Increased negative and reduced positive amygdala feedback on the insula was also observed in this study. A correlation between PTSD symptom severity and connectivity changes were shown when both PTSD and TENP group were included in a correlational analysis.

#### Functional Activity

Shin et al. presented stimuli (faces with different emotional expressions) to PTSD and TENP individuals (43). Significantly increased amygdala activity and decreased medial PFC activity were observed in the PTSD group when fearful facial expressions were presented. The degree of amygdala activity increase was correlated with the degree of medial PFC activity decrease, which was correlated with PTSD symptom severity. There was also a tendency for reduced habituation of amygdala activity in the PTSD group. An intervention study had policemen who had experienced trauma exposure undergo an fMRI scan while performing a memory task (44). Individuals with PTSD symptoms were subdivided into two groups, of which one received psychotherapy while the other was put on a waitlist for psychotherapy. Comparing scan results pre and post-psychotherapy revealed increased medial PFC activity and decreased amygdala activity in both the PTSD-psychotherapy group and the TENP group compared to the PTSD-waitlist group, where individuals still presented severe PTSD symptoms. A statistical connection was shown between imaging results and symptom severity. A more recent study included childhood abuse victims that were asked to perform a cognitive inhibition task while undergoing an fMRI scan (45). A statistical correlation was found between abuse severity and ACC activity in the PTSD group, suggesting that cognitive inhibition was significantly reduced in individuals with PTSD and severe abuse.

### Three-Group-Studies

In order to more reliably distinguish between genuine vulnerability factors and findings that are the result of trauma *per se* or other factors, more recent studies often include a control group of non-trauma-exposed, healthy subjects. Between-group comparison allows for a relatively reliable identification of resilience factors not associated with trauma exposure-related stress.

#### Structure

The very first study conducted as early as 1996 found hippocampal volume to be reduced in the PTSD group compared to TENP and control groups (46). However, hippocampal volume in this study was also correlated with the duration of war exposure, suggesting that reduced hippocampal volume might be either a vulnerability factor or a result of stress, or both. A study on women with a childhood history of sexual abuse confirmed the finding of reduced hippocampal volume in PTSD compared to TENP and control groups, with the difference being more pronounced between PTSD and control group compared to PTSD and TENP (47). A Gulf War veteran study also discussing potential epiphenomena, such as alcohol dependency or depressive disorder found a correlation of hippocampal volume with current PTSD symptom severity, but not with formerly diagnosed PTSD or current depressive episodes (48). Neither did this study observe an effect of age, number of additional traumatic life events, alcohol or cannabis dependency, or antidepressant medication on hippocampal volume. A study on burn victims suggests a size-reducing effect of stress on the hippocampus, finding smaller hippocampal volume in PTSD and TENP groups compared to controls but no differences between PTSD and TENP (49). Hippocampal volume was correlated negatively with burnt body surface, while it correlated positively with analgesic (and thus stress-reducing) medication with Ketamine. A number of additional studies were not able to replicate the above findings. No differences were found between hippocampal volumes of PTSD, TENP and control groups in populations of domestic violence victims (50), women with a history of childhood abuse (51), former prisoners of war (52), and holocaust survivors (53). As previously stated, certain epiphenomena need to be considered in the analysis of these results. One study on veterans demonstrated a selective volume reduction of the hippocampal head in the PTSD group but not a reduction of hippocampal volume, *per se* (54). A more recent study on adolescents with a history of abuse demonstrated increased hippocampal volume in the TENP group compared with both PTSD and control groups (55). Regarding the amygdala, studies investigating amygdala volume in populations of war veterans (46), domestic violence victims (50), and adolescents with a history of abuse (55) found no changes in amygdala volume for PTSD groups. However, the latter study reported a correlation of amygdala volume with PTSD symptom severity, as well as increased amygdala volume in the TENP group compared to PTSD and control groups (55). By contrast, one study demonstrated reduced ACC volume in the PTSD group of a study on refugees (56). ACC volume was also reduced in the TENP group compared to controls, yet to a much smaller degree. With respect to the PFC, one study on domestic violence victims found reduced PFC volume in both trauma-exposed groups compared to controls (50). More recent studies, contrarily, found a volume reduction of ventromedial PFC and orbitofrontal cortex in the PTSD groups of refugee (56) and childhood abuse victim populations (55) compared to TENP and control groups. In the refugee population, a slight reduction of ventromedial PFC volume was also observed in the TENP group.

#### Functional Connectivity

A study on war veterans found reduced default-mode network (DMN) connectivity, and increased salient network (SN) connectivity, especially with regards to increased amygdala-insula connectivity (57). There was also a significant increase in connectivity between DMN and SN networks. A study on war veterans demonstrated reduced connectivity between pgACC-PFC and pgACC-temporal lobe in both PTSD and TEMP groups compared to controls (58). Additionally, increased connectivity between rostral ACC and PFC was found in the TENP group. A follow-up study on the same population failed to demonstrate an effect of trauma-focused therapy on the above connectivity parameters, independently of therapeutic outcome (59). Contrarily, a study on adults with a history of childhood abuse did not replicate these results (60). An increase in ACC connectivity with occipital cortex regions was found, yet no changes in ACC connectivity with PFC, Amygdala, insula or core regions of other networks.

#### Functional Activity

One study found reduced neuronal activity, more specifically an increase in the number of inhibition-related mistakes during a task and a reduced recruitment of fronto-parietal brain areas (exclusive and reduced PFC activity), in the PTSD group compared to TENP and controls (61). These results were replicated in another study with participants undergoing an inhibition task while being MRI-scanned, with the task in the latter study, unlike the first, also including emotional components (62). The PTSD group again showed reduced PFC recruitment during the task, while an increased recruitment of fronto-temporal areas associated with conscious emotion regulation (“top-down control”) was observed in the TENP group. Another study on female sexual abuse victims asked to down-regulate their emotional reaction to negative images during a scan found a generally reduced PFC activity in trauma-exposed women (PTSD and TENP group) compared to controls (63). Upon emotion regulation, increased PFC recruitment was found in the TENP group compared to both PTSD and control groups.

### Twin Studies

This study design compares trauma-exposed individuals with PTSD symptoms and their non-exposed identical twin siblings to trauma-exposed individuals without PTSD symptoms and their non-exposed identical twin siblings. Using this study design, a number of factors can be reliably controlled for as genetic setup is identical between trauma-exposed and non-exposed groups. However, a number of lifestyle-related factors are nevertheless important contributors to potential differences found between twins, may interact with genetic factors and this needs to be accounted for in this design.

#### Structure

Analysis of hippocampal volumes of war veterans revealed a volume reduction in the PTSD group and their twins compared to TENP and their twins (11). The hippocampal volume of non-exposed twins of the PTSD group correlated with the PTSD symptom severity in the PTSD group, indicating strongly that reduced hippocampal volume is a vulnerability factor, rather than a result of exposure to stress. Other factors, such as alcohol dependency or major depressive disorder only had statistically significant effects on hippocampal volume in the PTSD group. The same research group later confirmed the above results and additionally found that specific characteristics of the PTSD group, such as increased vegetative reaction to trauma-associated stimuli, are not associated with the reduction in hippocampal volume (64). This is additionally confirmed by another study on war veterans finding reduced hippocampal volume in the PTSD group and their twins compared to TENP and their twins (65). Regarding other anatomical structures, a study on war veterans did not find any differences in amygdala volume between any of the groups, nor associations with psychopathological symptom severity (11). Reduced bilateral insular volume was found in the PTSD group and their twins compared to the TENP group and their twins (65). No differences in insular volumes were found between the respective twin groups. Finally, reduced pgACC volume was observed in a PTSD group and their twins compared to TENP and their twins (65). Additionally, a reduction of pgACC volume was also found in the PTSD group compared to their non-exposed twins, suggesting reduced pgACC volume might be both a vulnerability factor and a consequence of exposure to stress.

#### Functional Connectivity and Activity

To the best of our knowledge, no study investigated so far functional connectivity according to a twin-study design. Regarding activity, one study used a task reliably causing ACC activation during an MRI scan in war veterans (66). Increased dACC activity and increased response latency were observed in the PTSD group and their twins, suggesting increased ACC activation to be a vulnerability factor rather than a result of stress exposure based on these findings. The extent of ACC activation increase was correlated with the severity of clinical symptoms, but not with other comorbidities, such as depressive episodes or alcohol dependency.

### Longitudinal Studies

This study design examines trauma-exposed individuals immediately after the event and again at one or several follow-up time points. Parameters predicting the development of clinical symptoms are determined prospectively. Short-term effects of the traumatic event cannot be ultimately excluded in this design.

#### Structure

Hippocampus. Survivors of various catastrophic events were examined immediately after and again after a 6 months interval (67). Ten out of thirty-seven participants developed PTSD symptoms, but no difference was found between their hippocampal or amygdala volume and that of the TENP group for either time point. Contrarily, a more recent study involving 10 weeks of psychotherapy for trauma-exposed individuals suggests reduced hippocampal volume might be a vulnerability factor (68). Hippocampal volumes at the first measurement (i.e., before therapy started) were already significantly reduced in the group of individuals with persisting PTSD symptoms post-therapy compared to groups with TENP or PTSD with successful therapy. There were no differences in hippocampal volumes between the two latter groups.

#### Functional Connectivity and Activity

Presently, only one study has aimed at predicting clinical outcome immediately after trauma exposure based on connectivity patterns. In more detail, Zhou et al. examined 15 individuals 2 days after being exposed to a traumatic event and again 6 months later and found a negative correlation between amygdala-PCC connectivity and PTSD symptom severity after 6 months (69). To the extent of our knowledge, no study investigated so far potential associations between functional activity and resilience/vulnerability to stress in populations based on a longitudinal study design.

## Summary and Implications on the Neurobiology of Resilience

### Structure

The present state of the literature is relatively heterogeneous, yet especially 3-group-studies and twin studies, as well as prospective longitudinal studies allow for first conclusions to be drawn. Reduced hippocampal volume, relatively consistently present in PTSD individuals compared to TENP or controls, might be either a vulnerability factor or a consequence of stress exposure or both. It seems reasonable to assume a multifactorial genesis. Amygdala volume does not seem to be a vulnerability factor, nor were any changes described consistently following stress exposure. Reduced ACC, especially pgACC, and PFC volumes seem to be predisposing factors for increased vulnerability, while they are only moderately influenced by stress exposure. In terms of the neurobiology of resilience, unchanged ACC and PFC volumes and potentially to some extent reduced hippocampal volume are likely to be morphological indicators of resilience (see Table 1 for a detailed presentation of all discussed structural imaging studies).

### Functional Connectivity

Amygdala connectivity seems to be increased selectively in PTSD, potentially also predicting clinical outcome and symptom severity. Neuroanatomically, these findings seem plausible since an association is thus established between increased interaction of danger-detecting and emotional/cognitive/physical homeostasis-regulating regions on the one hand and increased risk of developing PTSD symptoms on the other hand. Equally importantly, increased DMN and SN connectivity and thus increased interaction between one network associated with self-referential activities, such as memory and daydreams and another network evaluating the importance of internal vs. external stimuli seems to be characteristic for individuals more at risk of developing PTSD symptoms following trauma exposure. Inversely, weak connectivity between danger-sensitive and self-referential networks might thus be a neurofunctional indicator of increased resilience (see Table 2 for a detailed presentation of all discussed functional connectivity imaging studies).

**Table 2:** Summary of functional connectivity findings.

**Authors**	**Study design**	**PTSD**			**TENP**			**HC**			**Results**
		***N***	**M/F**	**Age**	***N***	**M/F**	**Age**	***N***	**M/F**	**Age**	
Rabinak et al. (39)	2 groups	17	17M	30.12 ± 7.70	17	17M	33.71 ± 9.12	None			PTSD: Increased connectivity between amygdala and insula
Sripada et al. (40)	2 groups	15	15M	27.3 ± 4.5	14	14M	26.6 ± 3.3	None			PTSD: Increased connectivity between amygdala and insula, decreased connectivity between amygdala and ACC
Brown et al. (41)	2 groups	20	16:4	44.1 ± 11.0	22	16:6	44.0 ± 8.9	None			Increased connectivity between amygdala (BLA) and ACC/PFC in PTSD
Zhang et al. (42)	2 groups	33	12:21	52.06 ± 6.77	33	16:17	48.85 ± 6.39	None			PTSD: Increased connectivity between amygdala and PFC/hippocampus and decreased connectivity between mPFC and insula.
Sripada et al. (40)	3 groups	15	15M	27.3 ± 4.5	15	15M	26.6 ± 3.3	15	15M	26 ± 5.9	PTSD: Increased connectivity between amygdala, insula and ACC (SN), decreased connectivity between vmPFC and hippocampus (DMN), increased overall connectivity between DMN and SN.
van der Werff et al. (60)	3 groups	11	8/3	39.73 ± 9.61	11	8/3	40.36 ± 10.94	11	8/3	40.45 ± 9.47	Increased connectivity between dACC and bilateral lingual gyrus/occipital fusiform gyrus in TENP
Kennis et al. (58)	3 groups	31	31M	35.58 ± 9.66	25	25M	36.04 ± 10.15	25	25M	34.16 ± 9.32	Reduced connectivity between PFC and pgACC for PTSD and TENP, increased connectivity between PFC and rACC for TENP
Zhou et al. (69)	Longitudinal	15	11/4	41.52 ± 12.56	None			None			Connectivity between posterior cingulate cortex and amygdala/hippocampus at baseline predicted symptom severity after 6 months.

*Study design and study sample characteristics are presented for all studies assessing potential functional correlates of vulnerability/resilience to stress as assessed via resting-state fMRI. PTSD, post-traumatic stress disorder; TENP, trauma-exposed non-PTSD; HC, healthy controls; DMN, default-mode-network; SN, salience network*.

### Functional Activity

Based on the present literature, increased amygdala and ACC activities as a response to external stimuli are consistently described as characteristic features of individuals with increased vulnerability. Therapeutic interventions, such as trauma-focused psychotherapy seem to enable return of amygdala activity to normal levels. PFC activity, both as a response to external stimuli or through conscious modulation, seems to be of core importance. While reduced PFC activity appears to be characteristic for vulnerable individuals, TENP groups were shown to have increased PFC activity even compared to control groups. Since strong inhibitory effects of PFC on brain areas associated with emotion regulation have been described, it seems reasonable to assume an increased ability to exert cognitive control over emotional processes in resilient individuals. A recent study confirms this assumption, finding that PTSD individuals with increased dorsolateral PFC activity and decreased amygdala activity during an emotion regulation task prior to trauma-focused psychotherapy benefit significantly more from such therapy and achieve better symptom reduction (13). Additionally, the ability to consciously recruit brain areas associated with positive emotional experience during presentation of negative stimuli seems to have some importance for the neurobiology of resilience. Decreased activity in the amygdala/ACC and increased PFC activity during distinct tasks, particularly during neurocognitive processes associated with emotion-regulation in terms of top-down control mechanisms, may thus represent a neuro-functional correlate of increased resilience (see Table 3 for a detailed presentation of all discussed functional connectivity imaging studies).

**Table 3:** Summary of functional activity findings.

**Authors**	**Study design**	**PTSD**			**TENP**			**HC**			**Results**
		***N***	**M/F**	**Age**	***N***	**M/F**	**Age**	***N***	**M/F**	**Age**	
Shin et al. (43)	2 groups	13	13M	52.8 ± 7.3	13	13M	49.7 ± 8.9	None			PTSD: Increased activity in amygdala, decreased activity in mPFC, mPFC activity correlated with symptom severity (passive viewing of faces)
Peres et al. (44)	2 groups	12 and 12	12M/12M	31.2 ± 5.8 (PT) and 27.6 ± 3.9 (WL)	12	12M	28.2 ± 7.8	None			PTSD: Increased activity in amygdala, decreased activity in mPFC (memory task)
Stevens et al. (45)	2 groups	37	37F	35.4 ± 12.5	53	53F	41.1 ± 12.2	None			Correlation between activity in ACC and trauma severity (inhibition task)
New et al. (63)	3 groups	14	14F	38.7 ± 11.2	14	14F	38.5 ± 10.8	14	14F	31.7 ± 10.3	Decreased activity in PFC in PTSD, increased activity in PFC in TENP (emotion regulation task)
Blair et al. (62)	3 groups	14	2/12	33.9 ± 9.98	15	4/11	31.4 ± 7.94	19	2/17	32.4 ± 8.79	Decreased activity in PFC in PTSD, increased activity in PC in TENP (executive task)
Falconer et al. (61)	3 groups	23	13F, 10M	38.3 ± 12.16	23	13F, 10M	32.40 ± 15.00	17	6F, 10M	39.3 ± 12.6	PTSD: decreased activity frontoparietal (executive task)
Shin et al. (66)	Twin study	12 (twin pairs, i.e., one exposed and one unexposed twin)	12M	55.0 ± 2.9	14 (twin pairs, i.e., one exposed and one unexposed twin)	14M	56.4 ± 2.2	None			Increased activity in ACC for PTSD and their twins

*Study design, study sample characteristics and specific tasks are presented for all studies assessing potential functional correlates of vulnerability/resilience to stress as assessed via task-based fMRI. PTSD, post-traumatic stress disorder; TENP, trauma-exposed non-PTSD; HC, healthy controls; DMN, default-mode-network; SN, salience network*.

## Discussion

The present review aimed to investigate whether there are neurobiological correlates of resilience. Based on the data reviewed in this relatively recent area of research (1), a specific neurobiological correlate of resilience cannot be established, *per se*. A number of preliminary assumptions can be made on the basis of the reviewed above, however, which are discussed below.

First, there seems to be a spatial overlap between brain areas associated with increased resilience on the one hand and with emotion and stress regulation, on the other hand. Second, structural data suggest relatively consistently that increased gray matter volumes in ventromedial PFC, ACC (especially pgACC) and, to a lesser extent, hippocampus are associated with increased resilience, while amygdala morphology does not appear to play a vital role in this context. Third, decreased functional amygdala connectivity within the salience network, as well as decreased amygdala connectivity with default mode network structures seem to be associated with increased resilience. Fourth, more recent studies suggest an association of resilience with an increased ability to voluntarily recruit PFC and, to a lesser extent, ACC, suggesting a better “top-down” control due to the inhibitory effects of these brain areas on the amygdala. The latter findings provide options for future therapeutic interventions. One study demonstrated improved amygdala regulation through increased PFC influence in a neurofeedback-based MRI learning task in healthy individuals (15). Further research should explore whether such tasks can also prove beneficial in PTSD patients or as a preventive measure to improve resilience.

Resilience is a dynamic process of adapting to a significant and traumatic stressor that has to be investigated over time. Such a process of adaptation of a complex system will have neurobiological correlates itself. The study designs reviewed here, however, do not allow for a time-dependent description of neurobiological findings nor for the establishment of a causal relation between individual findings. The definition of inclusion and exclusion criteria is yet another challenge in the available literature. One issue is the definition of resilience as the absence of specific PTSD symptoms, with a large number of studies explicitly regarding individuals as resilient if they had other potentially trauma-related pathologies, such as depressive episodes or substance abuse disorders. Additionally, the number and types of traumatic experience vary greatly, as do other participant characteristics, such as age, gender, previous experience, etc., rendering between-study comparisons problematic. Yet another challenge is the diagnostic process, which itself is based on a categorical decision: if a certain number of PTSD symptoms is observed within a defined time period, a diagnosis is established. More recent approaches, such as the National Institute of Mental Health's concept of Research Domain Criteria, aim to develop trans-diagnostic systems to specifically match certain behavioral parameters and their neurobiological correlates at least for research purposes (70). This might lead to a shift from categorical systems toward trans-diagnostic, multidimensional inclusion criteria (71), which would potentially enable drawing conclusions between different study populations regarding findings on resilience.

Ideally, future studies would be based on longitudinal designs rather than cross-sectional ones. Participants should be recruited before (likely) traumatic exposure and should undergo multimodal examinations. Structural and functional neurobiological parameters should be determined in addition to detailed clinical assessment. Following traumatic exposure, during follow-ups and where applicable, following treatment, all physical and psychiatric comorbidities should be assessed along with the initially determined neurobiological parameters, allowing for the specific retrospective identification of clinical outcome predictors, as well as the demonstration of trauma- and therapy-associated changes.

Numerous other parameters can obviously influence the above observations. For example, genetic factors, such as a polymorphism of the gene encoding the catechol-O-methyl-transferase (COMT) can modulate the association between stress exposure and brain activity. One study demonstrates statistically significant associations between specific variations of this gene and increase or decrease in hippocampal activity, while associations between hippocampal activity and resilience are only shown in one group (72). Recent literature also increasingly demonstrates an increase in vulnerability when there is an attention shift toward negative stimuli, while a tendency toward prioritizing the processing of positive stimuli is associated with resilience (73). Additionally, there is increasing evidence for a gender-specific pattern of the described structural and functional changes: While male individuals largely present PFC, amygdala and hippocampus gray matter reductions following traumatic exposure, females often present with amygdala hyperactivity. This might not only explain the heterogeneity of study results, but also suggest far-reaching implications for the selection of adequate therapeutic measures (74).

## Conclusion

Understanding and furthering resilience-increasing factors through better describing vulnerability, including neuroimaging findings from a structural, functional connectivity and functional activity point of view, would be well-served in terms of treating and preventing PTSD. The above findings suggest that reduced hippocampal, anterior cingulate and prefrontal cortex volumes were associated with higher vulnerability. Furthermore, increased amygdala, default-mode and salience network connectivities were associated with higher vulnerability. Finally, increased amygdala and anterior cingulate cortex activities and decreased prefrontal cortex activity as a response to external stimuli were also associated with higher vulnerability, while increased prefrontal cortex activity was associated with lower vulnerability. Further research using suitable study designs is needed to better understand the underlying causalities and mechanisms.

## Author Contributions

ES, BK, and AM conceptualization of study concept/design; JB and AM literature screening; ES and BK quality control of data; JB, ES, BK, and AM data interpretation; JB manuscript preparation; ES, BK, and AM manuscript editing; JB, ES, BK, and AM manuscript review. All authors gave final approval of the version to be published and agree to be accountable for all aspects of the work in ensuring that questions related to the accuracy or integrity of any part of the work are appropriately investigated and resolved.

### Conflict of Interest Statement

The authors declare that the research was conducted in the absence of any commercial or financial relationships that could be construed as a potential conflict of interest.
